# Nutritional Management Mode of Early Cardiac Rehabilitation in Patients with Stanford Type A Aortic Dissection

This article has been retracted.

**DOI:** 10.1155/2022/2124636

**Published:** 2022-08-18

**Authors:** Lu Liu, Yongjian Yang

**Affiliations:** ^1^School of Public Health, Anhui Medical University, Hefei 230032, China; ^2^Department of Cardiovascular Surgery, First Affiliated Hospital of University of Science and Technology of China/Anhui Provincial Hospital, Hefei 230001, China

## Abstract

Malnutrition and metabolic disorders are common problems faced by patients with Stanford type A aortic dissection after surgery. Some patients have dietary problems such as malnutrition, unbalanced diet, and poor eating habits before surgery. Therefore, the nutritional management of early heart health can improve the nutritional support for perioperative recovery, to improve the pertinence. Therefore, active nutritional support after surgery will help to change malnutrition and metabolism and is of great significance to postoperative recovery and quality of life. This paper is aimed at studying the nutritional management mode of early cardiac rehabilitation in patients with Stanford type A aortic dissection. Based on the analysis of the pathogenesis of aortic dissection and the diagnosis of aortic dissection, two groups of patients were given individualized nutritional management scheme and routine nutritional scheme, respectively, and the nutritional risk differences between the two groups under different schemes were compared. The results showed that there was a statistical difference between the two groups at discharge. The NRS-2002 score of 14 cases in the observation group was less than 3 after nutritional intervention, indicating that there was no nutritional risk at discharge.

## 1. Introduction

There are many triggers for aortic dissection, and these triggers create voids in the middle layer of the aortic wall and into the bloodstream. If the blood is in a flowing state, the risk factor is relatively small, but if it is in a coagulated state, it can lead to catastrophic consequences. Because the patient is seriously ill, the mortality rate is particularly high, with aortic rupture as the main death. Data show that if aortic dissection surgery is performed within 48 hours of symptom onset, the mortality rate of patients is almost 50% [1, 2]. Among them, Stanford type A is the most severe type. Once found, it is recommended to carry out emergency surgery immediately. Due to the complicated operation process and the long duration of cardiopulmonary bypass, patients are prone to various postoperative side effects, and nursing care is troublesome and time-consuming. By doing a good job of postoperative follow-up treatment, the recovery rate of patients can be effectively improved [3, 4].

Aortic dissection is a local tear of aortic intima caused by various reasons, forming intimal rupture. The high-speed and high-pressure blood flow in the aortic cavity enters the mesentery through this fissure and separates it. The stripped intima and part of the mesentery gradually expand in the lumen to form intimal slices, separating the lumen from the true lumen and false lumen [5, 6]. The course of disease is acute aortic dissection within two weeks and chronic aortic dissection more than two weeks. There are two general classification methods of mezzanine, namely, Stanford classification and DeBakey classification. According to the degree of dissection involvement, Stanford classification is divided into Stanford type A involving the ascending aorta and Stanford type B not involving the ascending aorta [7, 8].

In recent years, with the progress of surgical technology, the treatment effect of Stanford type A aortic dissection has gradually improved, and the surgical mortality has gradually decreased [9]. However, Stanford type A aortic dissection surgery is difficult, and the incidence of postoperative complications is high. It is not enough to improve the therapeutic effect of Stanford type A aortic dissection surgery only by improving the surgical technology, but also need to use postoperative active nutritional support to change malnutrition and metabolism, so as to improve postoperative recovery [10–12].

Nutritional support has a long history, but it was not until the end of the twentieth century that it developed into an independent system. The significance of clinical nutritional support is not only the supply of nutrients but also the main means to improve the nutritional status of patients, such as treatment, maintenance of cell metabolism, and enhancement of immune function, but clinical efficacy. Some studies have also pointed out that the nutritional requirements of patients are also related to the prognosis of surgery [13–16]. Using scientific perioperative nutritional support to improve the physical vitality of high-risk patients has a good impact on improving the recovery cycle of postoperative patients, thereby reducing complications and shortening the duration of hospitalization [17, 18]. Patients undergoing acute abdominal resection due to stressful stimuli caused by eating dysfunction or the disease itself may be accompanied by huge nutritional deficiencies and potential low nutritional risks, coupled with severe postoperative injury and prolonged inability to eat; it can lead to many complications and poor prognosis such as hospitalization or long-term [19]. This problem can be effectively improved by carrying out scientific nutrition support planning. Scientific nutritional support can be carried out at the same time as the patient decides to operate, which can effectively shorten the patient's recovery period after surgery, and can play a very ideal intervention role even in the face of emergency patients [20, 21]. Excessive or insufficient nutritional support is not good for the body, and professional diet and nutritional risk assessment should be carried out before deciding whether to use nutritional support. The implementation of this step is the basis for scientific development of nutritional support and plays a significant role in reducing postoperative risks.

During the course of the research, the team collected and sorted out the existing research results in an all-round way, combined with the local hospital's experience in the diagnosis and treatment of aortic dissection, and selected 33 patients in the observation group with individualized nutritional management as the plan. For example, 32 patients in the control group were treated with routine nutrition management, and the differences in the rehabilitation of patients under different nutrition strategies were studied [22–25].

## 2. Nutritional Management Mode of Early Cardiac Rehabilitation in Patients with Stanford Type A Aortic Dissection

### 2.1. Pathogenesis of Aortic Dissection

#### 2.1.1. Hypertension

Among many factors, high blood pressure is one of the main reasons. Data show that the incidence of aortic dissection caused by hypertension accounts for about 70% of the total. If the patient has a long history of hypertension, the nutrients contained in the blood vessels will be gradually deficient, which will lead to the synthesis of elastic fibers, resulting in a decrease in elasticity [26, 27]. Increased stiffness and cystic necrosis of the aortic wall, weak areas, and subsequent dissection tendencies. If the blood pressure is too high, the shear pressure in the inner sheath increases, the inner sheath is more likely to rupture, and depending on the changes in the composition of the aortic wall, aortic dissection may form.

#### 2.1.2. Marfan Syndrome

Patients with Marfan syndrome are very rare and have a certain heritability. Patients may develop lesions in the connective tissues of the whole body such as the eyes and cardiovascular. However, the aortic dissection caused by it is the most serious harm of this sign. After dissection, it was found that this sign has a significant inhibitory effect on the formation of collagen, an important component of the blood vessel wall.

#### 2.1.3. Loeys-Dietz Syndrome

Loeys-Dietz syndrome is an autosomal dominant disorder of the connective tissue with common symptoms such as damage to blood vessels and bones. Similar to Marfan syndrome, it can also cause severe damage to the intimal structure of the aortic wall.

#### 2.1.4. Aortic Valve Bivalve Malformation (BAV)

BAV is more common in patients. The incidence of this congenital disorder is approximately 0.5-2%. Mainly manifested as cystic necrosis and lack of support, mainly following the degeneration of collagen and fibrous tissue in the central aorta, which eventually leads to rupture of the inner layer, leading to aortic dilatation and AD.

#### 2.1.5. Vascular Ehlers-Danlos Syndrome

The target of Ehlers-Danlos syndrome is also mainly connective tissue. In the current study, this symptom is divided into 6 subtypes, of which the vascular subtype is the most harmful.

### 2.2. Diagnosis of Aortic Dissection

#### 2.2.1. Digital Silhouette Angiography (DSA)

The oldest “gold standard” in the clinical treatment of aortic disease is cardiovascular angiography, but because of its invasiveness and high requirements for surgical techniques, it is inconvenient and increases the risk of AD in dangerous situations. Although DSA still retains its status as the “gold standard” for the treatment of aortic dissection, it has been largely replaced by CTA and is currently only used for endovascular repair and has not been used as a preoperative treatment option.

#### 2.2.2. Aortic CTA

At present, aortic CTA has become an important choice for rapid diagnosis of aortic dissection. With the continuous updating of imaging equipment, spiral CT 64 and 128 slices have a wide range of applications, the minimum slice thickness can reach 0.5-1 mm, the resolution is greatly improved, and the aortic bifurcation is joined. Powerful postprocessing software technology, such as 3D reconstruction technology, can clearly display the three-dimensional structure of the cardiovascular system, the degree of damage of the true and false lumen, and the location of the inner layer rupture, which helps to improve the grasp of the disease and is very useful for surgery [28, 29]. Due to its noninvasiveness and no limitation of metal bodies, it can completely replace DSA to a certain extent and provide further treatment guidance as a first-line diagnosis before open surgery or stent placement. In addition, convenient and economical examinations will be more easily accepted by patients, and it will be possible to establish regular postoperative monitoring mechanisms. The traditional use of CTA to monitor the changes in the process of peripheral residual false lumen and aortic remodeling has been widely used internationally, with potential observation of the effect of AD surgery. The disadvantage is that observing aortic insufficiency is not as good as ultrasound and requires injection of iodinated contrast agent, and people with renal failure are at risk of renal failure. In terms of diagnostic accuracy, the capture accuracy of CTA has reached more than 90%.

#### 2.2.3. Echocardiography (UCG)

UCG testing is fast, affordable, convenient, and noninvasive. The advantage is that critically ill patients can be checked in bed at any time to observe the condition of the aortic valve. However, this detection method has high requirements on the operator's experience and ability. The typical ultrasound change in AD is a ribbon reflex with varying degrees of normal pulse, where the innermost layer of the tear is wall-shifted during compression and cardiac-shifted during inflation. As seen in the arterial lumen, this is the breach where true and false lumens meet, so thrombi may also appear in the false lumen. Experienced physicians will judge the lesions of the blood vessel wall based on changes in blood flow rate. It may also occur with corresponding aortic valve insufficiency, pericardial hydrops, and occlusion of the aortic arch fan-shaped vessels. However, it is also affected by the patient's weight as well as other conditions. Transthoracic ultrasonography is simple and easy to perform, its sensitivity and professionalism are far lower than those of transesophageal ultrasonography, hypertension, etc., and usually requires anesthesia because it can aggravate the disease.

#### 2.2.4. Magnetic Resonance Imaging (MRI)

At present, MRI is the most accurate detection method. The disadvantage is that the test time is long, and the presence of metal in the body is the contraindication of the test. However, due to the highest soft tissue resolution of MRI in the medical field, Stanford type A patients can schedule MRI examination in advance. When there is metal in the patient's body, it can be considered to take out the metal before MRI examination [30]. Ad is shown as a double cavity on MRI. By comparing the space volume of the cavity, we can distinguish the true cavity from the false cavity. The patch in the coat shows a linear average signal between true and false double lumens. False lumen thrombus showed high signal intensity on T1WI and T2WI.

#### 2.2.5. Laboratory Diagnosis

Laboratory studies have shown that the vast majority of aortic dissection lesions are caused by vascular inflammation and destruction of vascular components. In recent years, research has mainly focused on early vascular endothelial injury, endothelial remodeling index, and inflammatory response index in AD patients. At this stage, the peripheral blood markers of AD patients are mainly divided into the following types. One is the main component test of the aorta. Elastin, like elastin, is another important component of the blood vessel wall. The second is the change in the measurement of various enzymes. The third is the research hotspot still under study, such as MMP and smooth muscle troponin.

## 3. Experiment

### 3.1. Research Objects

A total of 65 patients with Stanford A type were selected in this study. The patients were randomly divided into two groups for comparative study, as shown in Table 1. Among them, there were 33 cases in the observation group, including 20 males and 13 females, and 32 cases in the control group, including 17 males and 15 females. There was no statistical difference in the hospitalization conditions between the two groups (*p* > 0.05), indicating comparability.

### 3.2. Design a Nutrition Management Process

Nutritional support for patients with Stanford type A should be determined according to the specific characteristics of the patient's physical condition and blood analysis at different stages. One week or two weeks after the operation is set as an adjustment period, and a comprehensive analysis of the physical condition of the patients after the operation is performed as the basis for formulating the nutritional management process. Manage effectively according to the principles of routine nutritional care and pay attention to the individual phenomenon of insulin resistance and its metabolic characteristics in vivo. Malnutrition was corrected in a timely manner during the stressful period after surgery, and a reasonable calorie supply was provided according to individual characteristics. If it is 2-4 weeks after the operation, because the patient is also in the resynthesis stage of metabolism, the nitrogen metabolism level gradually becomes stable, and there is a reasonable nutrient guarantee, and the body protein gradually recovers. Fatty substances also begin to accumulate, and the body will slowly recover. At this stage, management will be implemented in a timely manner according to the principles of nutritional intervention, and the Stanford type A median artery and its risk factors will be gradually separated, and nutrition education will be strengthened to gradually establish the patient's complete nutritional structure, good eating habits, and self-administration ability.  Figure 1 shows the nutritional management process for 1-2 weeks after surgery.

### 3.3. Statistical Analysis

SPSS17.0 statistical software was used for analysis. Measurement data were described by means ± standard deviation ($\bar{X}\pm S$) (normal distribution), independent samples *t* test was used for comparison within the same two groups of time periods, and mean variance analysis of repeated measurement data was used for comparison at each time point within the same group. The chi-square test can also be used to describe the usage rate and composition ratio of enumeration data. *p* < 0.05 was regarded as the statistical significance of the difference.

A single population *t*-test tests whether a sample mean is significantly different from a known population mean. When the population distribution is normal, such as the population standard deviation is unknown and the sample size *n* < 30, then the dispersion statistic between the sample mean and the population mean is *t*-distributed. The test statistic is:

(1) $$\begin{array}{c} t=\frac{\bar{X}-\mu }{\sigma_{X}/\sqrt{n-1}}. \end{array}$$

If the sample is a large sample (*n* > 30), it can also be written as:

(2) $$\begin{array}{c} t=\frac{\bar{X}-\mu }{\sigma_{X}/\sqrt{n}}, \end{array}$$

where $\bar{X}$ is the sample mean.

## 4. Discussion

### 4.1. Result

As can be seen from Figure 2, the NRS-2002 scores of the two groups of patients before intervention were all >3 points, indicating nutritional risk. Most of the patients in the observation group and the control group scored 5 and 6 points, respectively. The composition ratio of NRS-2002 score before intervention between the two groups was not statistically different (*p* = 0.116), indicating comparability.

According to the data in Figure 3, there is a statistical difference between the two groups at the time of discharge (*Z* = −5.611, *p* < 0.05). Among them, the observation group and the control group scored 2 points and 4 points, respectively. The NRS-2002 score of 14 patients in the observation group was less than 3 after nutritional intervention, indicating that there was no nutritional risk at discharge.

### 4.2. Postoperative Intervention Strategies for Stanford Type A Aortic Dissection

#### 4.2.1. Family Intervention

Family intervention is a mode of intervention work carried out through the family members of patients. The family is in daily contact with the patient to better understand the patient's current recovery status, life expectancy, high demands, and aspirations. Family is the environment in which individuals live as a whole, which can provide patients with a sense of comfort that hospitals cannot provide. The mutual assistance of family members can help solve their psychological problems and improve the quality of life of patients after discharge. For example, in terms of sleep management of patients, in addition to the need for medical staff to regularly monitor patients with insomnia, pay attention to their sleep status. Hospitals can provide guidance manuals to help patient caregivers master the scientific methods of sleep intervention. If the patient nurses can cooperate in this work, it is very beneficial to adjust the patient's psychological state, which is very beneficial to the patient's recovery.

#### 4.2.2. Medication Compliance Intervention

Regardless of treatment, intensive care is required after surgery. During this period, drug use is an important part of the treatment process, which can play a vital role in the success or failure of the operation and the maintenance of the operation effect. For different patients, individualized drug delivery strategies should be developed. For example, for hypertensive patients, blood pressure control should be placed in a very important position. Emphasize the link between the disease and high blood pressure to the patient, and help the patient pay enough attention to the stability of blood pressure. Therefore, even after a patient is discharged from the hospital, blood pressure medication is required, even after successful surgery or invasive treatment.

#### 4.2.3. Health Education

At present, hypertension has been identified as the main influencing factor of dissecting aneurysm, and proper control of blood pressure can not only prevent the anatomy of the aorta but also prevent the recurrence of the aneurysm. Therefore, controlling blood pressure is crucial. Since blood pressure is affected by many factors, patients should pay attention to the fluctuation of blood pressure, monitor blood pressure with a sphygmomanometer at home, take antihypertensive drugs on time, and ask a specialist to adjust it regularly. During the early stages of withdrawal, patients should follow a bland, easily digestible diet. It is recommended to reduce sodium intake, engage in moderate activity, and avoid strenuous physical activity. For patients and their families, they love talking to doctors. However, it is not possible for nurses and physicians to teach specific patients for long periods of time in clinical practice. If patients want information from medical staff that will help them in their recovery, patients take certain actions, such as frequent visits to clinics, passing nursing homes, and frequent checks to see if medical staff are busy. Therefore, in this case, the department should regularly organize health education lectures, and organize specialized medical staff to give lectures to grouped patients. The training content includes daily life, eating habits, necessity of taking medicines, drug use, drug effects, and side effects.

#### 4.2.4. Psychological Counseling

In the early postoperative period, patients may feel anxious due to their unfamiliarity with the ICU environment, postoperative tracheal intubation, gastric tube, and intrathoracic drainage tube. Especially for patients with anatomical aneurysms and relatives who died of familial aneurysms, the psychological burden is heavier than other patients. Therefore, nurses using tubular beds should know the patient's genetic history of aneurysm dissection as early as possible before conducting psychological consultation. The long-term healing effect is also enough to let the patient know that the current science and technology have successfully cured the anatomical aneurysm. Additionally, it informs patients that the likelihood of anatomical recurrence after surgery is a low-probability event. At the same time, since high blood pressure is the main cause of aneurysm, blood pressure needs to be monitored after surgery, so the knowledge of aneurysm anatomy needs to be explained in more detail. Good blood pressure control has a positive effect on the prognosis and prevention of cardiovascular disease. It will influence and increase the patient's desire for discharge, a better life in the future, and confidence in recovery.

## 5. Conclusions

The situation of Stanford type A patients is complex, and there are many obstacles in the nutritional absorption of postoperative recovery. This situation has a negative impact on the postoperative recovery of Stanford type A patients. If we cannot formulate countermeasures as soon as possible, it will undoubtedly increase the postoperative risks faced by patients. Nutritional support can significantly promote the recovery of patients with Stanford type A aortic dissection. In order to better explore the establishment of nutritional support system for patients with this disease, this study proved the positive role of scientific nutritional support in improving the recovery effect of postoperative patients through experimental comparison. Based on the comprehensive collection and collation of the existing research results and combined with the hospital's experience in the diagnosis and treatment of aortic dissection, 33 patients in the observation group with individualized nutrition management as the scheme and 32 patients in the control group with routine nutrition management as the scheme were selected to study the rehabilitation differences of patients under different nutrition strategies. The results showed that there was a statistical difference between the two groups at discharge. The NRS-2002 score of 14 cases in the observation group was less than 3 after nutritional intervention, indicating that there was no nutritional risk at discharge. Finally, in order to better promote the postoperative recovery of patients with Stanford type A aortic dissection, this study also proposed the corresponding intervention countermeasures after Stanford type A aortic dissection. In the next research, this study will continue to adopt the method of group experiment to explore the formulation of nutritional support strategies for patients.

## Figures and Tables

**Figure 1:** Nutritional management process 1 to 2 weeks after surgery.

**Figure 2:** Comparison of preintervention NRS-2002 scores.

**Figure 3:** Comparison of NRS-2002 scores after intervention.

**Table 1:** Observation group and control group.

	Males	Females	Total
Observation group	20	13	33
Control group	17	15	32

## Data Availability

The data used to support the findings of this study are available from the corresponding author upon request.

## References

[1] Klassen S. L., Hutchison S. J. (2019). Quadricuspid aortic valvulopathy and acute type A aortic dissection. *ACI Open*.

[2] Pan X., Lu J., Cheng W., Yang Y., Zhu J., Jin M. (2018). Independent factors related to preoperative acute lung injury in 130 adults undergoing Stanford type-A acute aortic dissection surgery: a single-center cross-sectional clinical study. *Journal of Thoracic Disease*.

[3] James B., Kelsey U., Arjuna P. (2018). Cold agglutinin disease complicating management of aortic dissection. *Transfusion & Apheresis Science*.

[4] Dumfarth J., Kofler M., Stastny L. (2018). Stroke after emergent surgery for acute type A aortic dissection: predictors, outcome and neurological recovery. *European Journal of Cardio Thoracic Surgery Official*.

[5] Wu J. T., Sun Q., Wang Y. (2019). Effect of preoperative symptomatic pericardial effusion on postoperative rehabilitation of patients with Stanford type A aortic dissection. *South China Journal of Defense Medicine*.

[6] Li Z., Meng W. X., Kang K. (2020). Research progress in the prevention and treatment of postoperative hypoxemia in patients with Stanford type A aortic dissection. *China Cardiovascular Disease Research*.

[7] Lu L., Zhou X. D., Wang J., Wu Y. B., Huang W. C., Xie Q. L. (2022). Study on risk factors of postoperative delirium in patients with Stanford type A aortic dissection. *Zhejiang Medical Journal*.

[8] Shi H. P., Wang X. Z., Yang X. J. (2017). Retrospective study on the risk factors of postoperative acute renal injury in patients with acute Stanford type A aortic dissection. *Chinese Journal of Critical Care Medicine*.

[9] Li Y. L., Zhao Y. L., Li Y. C. (2019). Nursing study on postoperative complications of patients with acute Stanford type A aortic dissection. *Capital Food and Medicine*.

[10] Wang W. X., Xu X., Wang W. (2019). Comparison between Stanford type A aortic dissection combined surgery and aortic arch replacement stent "elephant trunk" surgery. *Chinese Journal of Thoracic and Cardiovascular Surgery*.

[11] Zheng Q. (2020). Effect of 4R crisis management on preventing postoperative delirium in patients with Stanford type A aortic dissection. *Journal of Qiqihar Medical College*.

[12] Cheng Y. Z., Tao L., Liu Y., Huang W. Q., Zhu T. J. (2005). De Bakey type I and II aortic dissection surgery, postoperative rehabilitation and mid-term follow-up. *Chinese Journal of Cardiovascular Disease Research*.

[13] Zhang Z., Cui F., Cao C., Wang Q., Zou Q. (2022). Single-cell RNA analysis reveals the potential risk of organ-specific cell types vulnerable to SARS-CoV-2 infections. *Computers in Biology and Medicine*.

[14] Yan J., Yao Y., Yan S., Gao R., Lu W., He W. (2020). Chiral protein supraparticles for tumor suppression and synergistic immunotherapy: an enabling strategy for bioactive supramolecular chirality construction. *Nano Letters*.

[15] Zhuo Z., Wan Y., Guan D. (2020). A loop-based and AGO-incorporated virtual screening model targeting AGO-mediated miRNA–mRNA interactions for drug discovery to rescue bone phenotype in genetically modified mice. *Advanced Science*.

[16] Li H., Wang F. (2021). Core-shell chitosan microsphere with antimicrobial and vascularized functions for promoting skin wound healing. *Materials & Design*.

[17] Yuan P. J., Wong W. K. (2018). Acute myocardial infarction and concomitant stroke as the manifestations in a patient with type A aortic dissection: a case report with three years of follow-up. *Acta Cardiologica Sinica*.

[18] Takagi H., Ando T., Umemoto T. (2018). Meta-analysis of seasonal incidence of aortic dissection. *American Journal of Cardiology*.

[19] Zhang L., Zhou J., Jing Z. (2018). Glucocorticoids regulate the vascular remodeling of aortic dissection via the p38 MAPK-HSP27 pathway mediated by soluble TNF-RII. *eBioMedicine*.

[20] Li G., Li P., Liu S., You B. (2022). Follow-up of robotic mitral valve repair: a single tertiary institution experience in China. *Computational and Mathematical Methods in Medicine*.

[21] Miyairi T., Miyata H., Chiba K. (2018). Influence of timing after thoracic endovascular aortic repair for acute type b aortic dissection. *Annals of Thoracic Surgery*.

[22] Cao Z., Wang Y., Zheng W. (2022). The algorithm of stereo vision and shape from shading based on endoscope imaging. *Biomedical Signal Processing and Control*.

[23] Xu Q., Zeng Y., Tang W. (2020). Multi-task joint learning model for segmenting and classifying tongue images using a deep neural network. *IEEE Journal of Biomedical and Health Informatics*.

[24] Obireddy S. R., Lai W. (2021). Multi-component hydrogel beads incorporated with reduced graphene oxide for ph-responsive and controlled co-delivery of multiple agents. *Pharmaceutics*.

[25] Ji X., Hou C., Gao Y., Xue Y., Yan Y., Guo X. (2020). Metagenomic analysis of gut microbiota modulatory effects of jujube (Ziziphus jujuba Mill.) polysaccharides in a colorectal cancer mouse model. *Food & Function*.

[26] Sultan I., Siki M. A., Bavaria J. E. (2018). Predicting distal aortic remodeling after endovascular repair for chronic DeBakey III aortic dissection. *The Annals of Thoracic Surgery*.

[27] Qiu J. T., Zhang L., Luo X. J. (2018). Correlation between of aortic dissection onset and climate change. *Chinese Journal of Surgery*.

[28] Zhang Z., Wang L., Zheng W., Yin L., Hu R., Yang B. (2022). Endoscope image mosaic based on pyramid ORB. *Biomedical Signal Processing and Control*.

[29] Liu S., Yang B., Wang Y., Tian J., Yin L., Zheng W. (2022). 2D/3D multimode medical image registration based on normalized cross-correlation. *Applied Sciences*.

[30] Brunet J., Pierrat B., Badel P. (2021). A parametric study on factors influencing the onset and propagation of aortic dissection using the extended finite element method. *IEEE Transactions on Biomedical Engineering*.

